# Analysis of Nursing Effect of Comprehensive Nursing Intervention on Hemodialysis Patients with Uremia

**DOI:** 10.1155/2022/5820707

**Published:** 2022-09-26

**Authors:** Lanfang Hu, Yanting Ma, Lihong Wang, Yapping Dai

**Affiliations:** Hemodialysis Room of Suzhou Hospital of Integrated Traditional Chinese and Western Medicine, Suzhou 215101, Jiangsu, China

## Abstract

Uremic pruritus affects 50–90% of hemodialysis patients, making it one of the most frequent medical issues among this group. Pruritus can lead to skin infections, desquamation, pathological skin changes, sleep problems, anxiety, depression, and social problems. The epidemic of uremia pneumonia has put a lot of stress on hemodialysis patients, resulting in negative feelings. As a result, during the prevention and control of uremia, rigorous management and improved nursing intervention are critical. During the uremia disease outbreak, this study will examine and assess the impact of clinically refined nurse intervention on patients receiving maintenance hemodialysis.

## 1. Introduction

End-stage renal disease requires hemodialysis as a conventional therapy (ESRD). The number of hemodialysis patients grew from 41,905 in 2005 to 45,894 in 2007, according to recent research by the National Kidney Foundation (ROC (2007)) [1]. According to the study, sleeplessness, exhaustion, muscular discomfort, muscle spasms, and dry skin are common symptom in hemodialysis patients, all of which can significantly impact their life satisfaction [2].

Patients undergoing hemodialysis are between 50 and 90 % likely to be affected by it [3]. In a study conducted in Taiwan on hemodialysis patients in 2003, two-thirds of respondents reported experiencing pruritus symptoms on a daily basis, and 45% of respondents said they had pruritus for more than six months [4]. Another research of hemodialysis patients discovered that most pruritus medications were unsuccessful [5].

Pruritus can increase the risk of skin infections, desquamation, and degenerative changes of the skin. Insomnia, anxiety, sadness, and social dysfunction are among the other difficulties [6]. It has been observed that hemodialysis patients who suffer with pruritus may get relief from it via the use of aromatherapy, acupressure, UV ray treatment, acupuncture, and primrose oil applications [7]. Nevertheless, the actual deployment of such therapies is restricted because of the high cost and/or complexity of these interventions. This research investigated a straightforward treatment for itchy skin that can be applied at home by hemodialysis patients without the assistance of a medical professional. The treatment involves the use of regular baby oil and works by preventing the transmission of nerve impulses that are irritating.

Pruritus seems to be the most common skin symptom seen in patients with end-stage renal illness (ESRD), and it may be very irritating for patients who are receiving dialysis [8]. Patients who have reached the terminal stage of renal disease, especially older patients, seem to have dry skin. Pruritus affects 37–90% of hemodialysis patients in Taiwan. The frequency of pruritus reported in response to the length of hemodialysis treatment varies depending on the study's duration. According to one study, 815 % of patients with hemodialysis had itchy skin during the first stage of treatment. In yet another study of hemodialysis patients in Taiwan, the researchers found that the majority of patients experienced pruritus within the first 3 months, 839% of patients suffered itching within the first 6 months, 322% of patients encountered pruritus symptoms weekly, and 677% of patients suffered dermatitis herpetiformis symptoms daily. Additionally, the researchers found that the majority of patients suffered itching within the first three months of treatment. The majority of patients develop pruritus between the 3rd and 12th month after starting hemodialysis, and 875% of patients continue to have it after receiving medical therapy. It was also revealed that 43% of hemodialysis patients had pruritus for six months in a row. The complete body was harmed in 555% of the cases, the abdomen in 278%, and the limbs in 167% of the cases. In another research, 258% of hemodialysis patients reported a hot feeling in the afflicted region, 226% claimed ache, and 516% just reported itching. The afflicted region is generally symmetrical, and the itching can be even severe than mosquito bites [8]. On the other hand, the pruritus that this patient group experiences is typically classified as moderate to severe. In order to provide more effective treatment, it is thus essential to determine the underlying processes and factors that contribute to pruritus.

## 2. Pruritus Mechanisms and Associated Causes

Because pruritus is caused by activation of the “C nerve fibres,” also referred to as “itch fibres,” and stopping their transmission lowers itching [9]. On the surface of the skin, the terminal points of free amyelinic lines are where you will find itch receptors. Itching receptors provide signals to a spinal dorsal horn, which are subsequently carried to the cerebral cortex via the spinothalamic tract's so-called “amyelinic C nerve impulses.” This causes the sense of itching and the need to scratch [10].

Dialysis is an essential treatment for people who have chronic renal illness because it extends the amount of time they are able to live and improves their quality of life [11]. The human body may be helped to get rid itself of waste products that are harmful and poisonous via the process of dialysis [12]. On the other hand, patients who do not comply with their treatment may have an undesirable consequence [13]. If, for example, patients carefully monitor their daily food and fluid intake, this might lead to an increase in the amount of excretion power needed, which in turn can cause pulmonary edema, bone demineralization, metabolic imbalance, cardiovascular injury, and death [14].

It is generally acknowledged that nursing engagement is more crucial in enhancing patients' conformity with their dialysis treatment. Education, training, and behavioral changes that assist patients in acquiring a better knowledge of dialysis and adopting healthy living habits have been shown to increase patient conformity with the treatment [15, 16]. Few studies have explicitly tested conformity and published the conformity rate [17]; however, the interdialytic weight gain (IDWG) and serum phosphorus level are the most often reported indicators for complete conformance. Conformity requirements have been published by the WHO [18].

Conformity measures are generally inconsistent in general [19]. Some studies, for example, show biomarker changes after the intervention that contradict clinical outcomes. For the purpose of this meta-analysis, we conducted a literature review to determine the impact that nurse intervention has on dialysis conformity. Additionally, our findings included conformity and nonconformity with qualitative indicators and clinic significance.

## 3. Background

### 3.1. Nursing Intervention Techniques

Nursing interventions are actions a nurse takes to implement their patient care plan, including any treatments, procedures, or teaching moments intended to improve the patient's comfort and health. These actions can be as simple as adjusting the patient's bed and resting position—or as involved as psychotherapy and crisis counseling. While some nursing interventions are doctors' orders, nurse practitioners can also develop orders using principles of evidence-based practice. Common nursing interventions include the following:

- Bedside care and assistance
- Administration of medication
- Postpartum support
- Feeding assistance
- Monitoring of vitals and recovery progress

A nursing rationale is a stated purpose for carrying out nursing intervention. Nursing interventions are actions that nurses perform to help patients achieve specified health goals. A nursing rationale is written next to each nursing intervention in the nursing care plan.

Closely observe the elderly patients with severe pneumonia in general, such as vital signs and the indicators. The patient's condition to conduct a comprehensive assessment of the risk factors may occur to exclude the indicators, such as whether hypoxemia, with or without high carbon dioxide, and so on. Ventilation dysfunction, the body hypoxia occurs, the patient may have respiratory symptoms such as changes in symptoms, so in daily care, they should pay attention to abnormal breathing frequency. The main manifestations of septic shock for blood pressure and body temperature decreased, so in patients with blood pressure, decline in body temperature should be considered due to septic shock. Patients with severe brain tissue hypoxia, ischemia, or carbon dioxide retention generally present with early abnormalities. Therefore, the early detection of patients with changes in condition should be promptly reported to the attending physician and as soon as possible to deal with to prevent the occurrence of critical illness.

In the treatment of elderly patients with severe pneumonia in patients with the humidification respirator treatment process, the respiratory tract care is also important. Respiratory tract management mainly includes the following four parts, namely, continuous respiratory tract humidification, drug ultrasonic atomization, auxiliary shot back expectoration, effective sputum suction, and so on. First is the continuous respiratory tract wetting process. Elderly patients with severe pneumonia due to infection and other factors have a series of respiratory symptoms, such as mucinous secretions; decreased respiration or arrest of tracheal mucosal ciliary movement; Phlegm is difficult to cough out and even form phlegm plug; difficulty breathing due to obstruction of the respiratory tract; purple lips, and so on. The application of humidifier enhanced the patient's respiratory tract clearance ability and help to cure patient in certain degree at the same time. In the clinical practice, humidifier gradually replaced the conventional way of humidification, due to simple operation and highly effective features.

The study group got psychological nursing that was based on the treatment group that was given to the treatment group. Standard hemodialysis nursing was provided to the treatment group. Prior to, during, and after dialysis are the three points at which psychological nursing is evaluated. Before beginning dialysis, there should be clear and open communication between patients and their doctors. Additionally, the patient's mental state and their psychological requirements should be well understood. Before delivering psychological therapy to a patient who was not in a good mood, the nurse should first participate in active dialogue with the patient, listen calmly, and discover the reasons of the patient's low mood. It is important for patients with diabetes and uremia who have never seen a doctor to be given a full assessment of the illness by their nurse. As a result, the patients will have a better grasp of their condition, and they will be less frightened about hemodialysis. When presenting essential information about hemodialysis as well as concerns during dialysis, it is necessary to use appropriate languages or dialects. This is necessary in order to accommodate the wide range of cultural backgrounds represented among patients [20, 21].

During the dialysis process, it is important to be aware of the numerical deviation of the dialysis machine as well as any changes in the patient's vital signs in order to notice the patient's suffering in a timely way. Furthermore, the nurse should routinely visit the patients and inquire about their thoughts, offer them advice on proper posture, and engage them in updateable suggestible discussion to validate their existence.

On the one hand, patients will have something to do, which will divert their attention and reduce the discomfort caused by hemodialysis. Patients on hemodialysis having uremia must be issued a disease-related newspaper, booklet, or periodical so that they may learn about their illnesses and acquire disease-resistant confidence. After dialysis, the nurse should assist the patients in getting clothed, inquire about any discomfort, and advise them to relax. If there is no discomfort, the patients will also be ready to travel. Communication with elder relatives should always be focused on the psychological requirements of the patient, so that the patient may acquire concerns that are timely and appropriate from relatives. And, since these worries are frequently expressed in some aspects of life, addressing them may greatly enhance a patient's confidence, which not only functions as a psychological signal but also has a considerable bearing on the therapeutic process.

Maintenance hematodialysis (MHD) is an important substitution therapy for chronic end-stage renal disease (ESRD). Since MHD treatment is long term and mainly based outside of a hospital setting, reasonable and correct nursing interventions are very important. Patients with uremia usually exhibit very poor residual renal function and a variety of complications, such as malnutrition, severe anemia, infection, and dysfunction of the heart, lung, and liver and other organs, among other problems (Figure 1).

## 4. Psychological Assessment Techniques

Both the self-rating anxiety scale (SAS) and self-rating depression scale (SDS) were applied in this study. Patients undergoing hemodialysis who also had uremia were given the SAS in order to evaluate their psychological well-being. With the help of the SPSS 16.0 software program and the mean value standard deviation, the statistical analysis was carried out (*x s*). An independent sample *t*-test and paired *t*-test were applied to contrast the pre- and posttreatment findings for every group. A paired *t*-test was used to compare the results of each group prior to and after therapy. The examining efficiency must be less than 0.05, which is the given threshold.

Let

(1) $$\begin{array}{c} f:\left[a,b\right]⟶\mathbb{R}, \end{array}$$

be a continuous function on the closed interval[*a*, *b*], and differentiable on the open interval (*a*, *b*), where *a* < *b*. Then, there exists some *c* in (*a*, *b*) such that

(2) $$\begin{array}{c} f^{\prime }\left(c\right)=\frac{f\left(b\right)-f\left(a\right)}{b-a}. \end{array}$$

As an extension of Rolle's theorem, it is known as the mean value theorem:

(3) $$\begin{array}{c} f\left(a\right)=f\left(b\right). \end{array}$$

As a result, the value on the right-hand side is zero. In a broader context, the mean value theorem is still true. for every *x* in (*a*, *b*), the limit

(4) $$\begin{array}{c} \underset{h⟶0}{\text{lim}}\frac{f\left(x+h\right)-f\left(x\right)}{h}, \end{array}$$

is defined as a number that is either equal to finite or infinite. It is important to note that the theorem, in its given form, is invalid if the values of a differentiable function are complex rather than real. For example, define

(5) $$\begin{array}{c} f\left(x\right)=e^{xi}, \end{array}$$

for all real *x*. Then,

(6) $$\begin{array}{c} f\left(2\pi \right)-f\left(0\right)=0=0\left(2\pi -0\right). \end{array}$$

While

(7) $$\begin{array}{c} f^{\prime }\left(x\right)\neq 0. \end{array}$$

These mathematical assertions are referred to as Lagrange's mean value theorem (Figure 2).

Let *μ* stands for the mean of random variable *X* with density *f*(*x*):

(8) $$\begin{array}{c} \mu \equiv \text{E}\left[X\right], \end{array}$$

where

(9) $$\begin{array}{c} E\left(x\right)=\overset{+\infty }{\underset{-\infty }{\int }}xf\left(x\right)\text{ d}x. \end{array}$$

The STD *σ* of *X* is expressed as

(10) $$\begin{array}{c} \sigma \equiv \sqrt{\text{E}\left[{\left(X-\mu \right)}^{2}\right]}. \end{array}$$

Therefore,

(11) $$\begin{array}{c} \sigma ==\sqrt{\overset{+\infty }{\underset{-\infty }{\int }}{\left(x-\mu \right)}^{2}f\left(x\right)\text{ d}x}, \end{array}$$

which may be shown to be equivalent (see Figure 3):

(12) $$\begin{array}{c} \sqrt{\text{E}\left[X^{2}\right]-{\left(\text{E}\left[X\right]\right)}^{2}}. \end{array}$$

The standard deviation is calculated as follows: when *X* selects random values from a finite data set consisting of *x*_1_, *x*_2_,…, *x*_*N*_, where each value has the same probability: $\sigma =\sqrt{1/N\left[{\left(x_{1}-\mu \right)}^{2}+{\left(x_{2}-\mu \right)}^{2}+\cdots +{\left(x_{N}-\mu \right)}^{2}\right]},\;$ where

(13) $$\begin{array}{c} \mu =\frac{1}{N}\left(x_{1}+\cdots +x_{N}\right). \end{array}$$

Or, by using summation notation,

(14) $$\begin{array}{c} \sigma =\sqrt{\frac{1}{N}\overset{N}{\underset{i=1}{\sum }}{\left(x_{i}-\mu \right)}^{2}}, \end{array}$$

where

(15) $$\begin{array}{c} \;\mu =\frac{1}{N}\overset{N}{\underset{i=1}{\sum }}x_{i}. \end{array}$$

If, rather from having probabilities that are equal, the values have different probabilities, then we will say that *x*1 has the probability *p*1 and *x*2 has the probability *p*2,…, *pN* is the chance that *xN* will occur. The standard deviation, in this particular instance, will be equal to

(16) $$\begin{array}{c} \sigma =\sqrt{\overset{N}{\underset{i=1}{\sum }}p_{i}{\left(x_{i}-\mu \right)}^{2},} \end{array}$$

where

(17) $$\begin{array}{c} \mu =\overset{N}{\underset{i=1}{\sum }}p_{i}x_{i}. \end{array}$$

The STD of a continuous real-valued random variable *X* with the probability density function *p*(*x*) is

(18) $$\begin{array}{c} \sigma =\sqrt{\underset{X}{\int }{\left(x-\mu \right)}^{2}\;p\left(x\right)\text{ d}x}, \end{array}$$

where

(19) $$\begin{array}{c} \mu =\underset{X}{\int }x\;p\left(x\right)\text{ d}x. \end{array}$$

Figure 4 depicts an example of the same mean but various standard deviations. The red and blue populations' averages and standard deviations are 100 and 50, respectively.

Baby oil has antipruritic properties.

By using baby oil, which contains a combination of hydrating virgin coconut oil and mineral oil, sufferers of neurosis and desquamation see a reduction in their symptoms. Baby oil that has been refrigerated may minimize inflammation as well as chemical sensitivity by preventing the passage of nerve signals along the C nerve fibers. The effects of cold temperatures include constriction of the blood vessels, a slowing of cell metabolism and nerve transmission, disruption of the transmission of nerve fibers, paralysis of neural receptors, and numbing of the treated area [22].

### 4.1. Important Things to Remember While Using Cooled Baby Oil

The oily solution's temperature should usually be 15°C [21]. Kennet et al. (2007) made the shocking discovery that the optimal temperature range for human skin is 10 to 15 C that is 5 degrees cooler than the commonly suggested range. According to their findings, cold treatment, through reducing skin temperature, has a calming impact on the skin, according to their findings. According to the recommended application method, baby oil should be administered to the afflicted region for 15 to 20 minutes, but not for more than thirty minutes at a time. [21] recommend a 30–60-minute interval between cold treatments. However, if the patient experiences pain, the cold treatment should be discontinued.

Chilled (10–15 C) and unchilled (24–26 C) baby oil were the tested interventions. Mineral oil and fragrance were the only components in the infant oil employed in this investigation. The baby oil preparations were hidden from all participants. The study procedure is listed in Table 1. After informing the experimental groups that they were going to be tested, either cold or room temperature baby oil had to be applied for 15 minutes at least once every day. Papers with which to make a record of the date and time of each event application were made available.

## 5. Methods

### 5.1. Queries and Datasets

In the databases PubMed, Cochrane, and Embase, we looked for the following keywords, which led us to the discovery of original research papers (from 2000 to 2016, a total of 190 months). (Dialysis, renal disease, hemodialysis, kidney) AND (conformity, IDWG, adherence, serum phosphorus) AND (nursing, intervention, care). The year was selected as a starting point since that point had significantly modified the conformity standards; prior to the year 2000, the majority of study designs and quality were subpar.

The following criteria would be used in the selection process: (I) population: patients with final renal dysfunction who received either hemodialysis or peritoneal dialysis at the same time in a nursing home or hospital; (ii) the involvement was a cognitive, educational, and/or attitudinal oral or video intrusion delivered by caregivers or nurses; (iii) the comparative involvement was a standard treatment regulation; (iv) the performance indicators were IDWG, conformity, nonconformity, and phosphorus; and (v) the design of this study was (RCT).

### 5.2. Information Extraction and Evaluation

Each study included documentation of the primary author, the year the publication was made, the sample size, the research methodologies, and the result measures. To determine eligibility, two investigators independently retrieved data as well as trial quality characteristics from the papers chosen for inclusion in the meta-analysis. An independent third party investigator analyzed the retrieved data by importing it into a standardised Excel file. Any differences were handled by discussion and agreement. The rate of conformity/nonconformity, as determined by the Department Of Health, was the outcome measurement.

The sample size of the trials ranged from 15 to 220 (a total of 817 patients, 429 males and 388 females). The patients were mainly from China, the USA, and the UK and thus represented Asia, Europe, and Northern America to eliminate regional confounding. Although the intervention methods utilized in the experimental group were inconsistent, all interventions were provided by professional nurses. The Jadad score ranged from 3 to 4.

The Jadad scale was utilized so that we could determine the amount of methodological complexity that was demonstrated by each experiment. In randomized controlled trials (RCTs), the scale consists of three categories: randomization (ranging from 0–2 points), blinding (ranging from 0–2 points), and dropouts and withdrawals (ranging from 0-1 point). Each of the points is given a one-point rating. When the technique of randomization and/or blinding is provided and is suitable, another point is awarded; when it is not, a point is subtracted. As a consequence of this, the quality scale ranges from 0–5, with higher ratings representing more accurate reporting. When the Jadad score is 2, the studies are deemed to be of poor quality; however, when the number is 3, the results are considered to be of good quality [19]. This investigation adhered to the suggested form of reporting, which is referred to as the declaration items for observational studies and meta-analyses [20].

### 5.3. Analysis of the Data

For the purpose of combining all of the data, RevMan 5.3.0 (http://ims.cochrane.org/revman) was used. The conformity rates were calculated based on the available research. Even after contacting the authors through e-mail, there were a few instances in which the conformity rate was not clearly mentioned in the literature and could not be established in any way, shape, or form. As a consequence of this, we computed it by using a complex statistical simulation under the assumption that either the IWDG or the serum phosphorus distributions are normal. Following that, the conformity rate was computed by using the “NORM.DIST” function included in the Microsoft “Excel” software and basing it on the aforementioned standards. Extracted results were based on the major endpoint time point in each of the included studies or, if no primary endpoints were provided, on the characteristics of patients at their most recent visit. In the end, both the relative differences (RD) and the pooled RD were taken into consideration when coming to a judgment. Since the investigator included patients who satisfied the nonconformity condition and interfered in particular tests, a random effects model was applied. In the meanwhile, the researcher included patients into the study who did not comply with the requirements. Nonetheless, there were authors who participated in the research who included all CKD patients who were on dialysis. As a direct result of this, when we assumed that the baseline in a specific trial was balanced, RD was a more trustworthy statistic than OR did. In addition to that, we carried out a sensitivity analysis on OR and then published the findings. The *I*2 statistic, which is a quantification of disagreement between research, was utilized in order to examine the degree to which investigations were diverse. This was done to see whether there was a substantial distinction between the trials. Low heterogeneity was classified as having an *I*2 of 25 to 50%, medium heterogeneity as having an *I*2 of 50% to 75%, and high heterogeneity as having an *I*2 of >75%. If the value of *I*2 was more than 50%, sensitivity analyses were performed in order to identify possible sources of heterogeneity. These analyses consisted of omitting one study at a time and determining the effect that each study had on the overall pooled estimate. We carried out an analysis of the data in subgroups depending on the various time periods. Any apparent publishing bias was uncovered by a visual examination of the Begg funnel plots. The threshold of significance was determined to be *p* 0.05.

## 6. Results

The first search turned up 88 articles that were pertinent, but based on their titles and abstracts, we were able to determine that 64 of them were not relevant because they included duplicate research, reviews, or other sorts of publications (See Figure 5). Twenty-four studies were identified as possibly relevant. Two were elected for full-text examination, while two were not. 13 were eliminated due to lack of vital information. For research purposes, nine RCT studies were finally chosen, six of which were published in English and three were published in Chinese.

## 7. Characteristics of Inquiry

Table 2 summarizes the key features of the nine research published between 2003 and 2016. The studies' sample sizes ranged from 15 to 220 participants (for a total of 817 people, 429 men and 388 women). The patients were primarily from China, the United States, and the United Kingdom, representing Europe, Asia, and Northern America to avoid regional confusion. Despite the fact that the study group's intervention approaches were uneven, all treatments were administered by professional nurses. Jadad's rating went from 3 to 4.

## 8. Meta-Analysis of Outcome Measures

It was found that nursing involvement was significantly associated with the increased higher rate of dialysis conformity (relative risk 0.15, 95% confidence interval (CI) 0.071–0.231, *p* = 0.00031, for heterogeneity, *I*2 = 44%, *p* = 0.017; odds ratio 2.171, 95% confidence interval (CI) 1.381–3.421, *p* = 0.0008, for heterogeneity; Figures 6 and 7). According to the results of the RD study, patients who got nursing help showed higher conformity with their dialysis treatments by 15% compared to those who received standard medical care.

Patients who received additional nurse assistance had almost 2-fold greater chances to comply with dialysis than those who received standard care, according to sensitivity analysis, which corroborated the results found for RD. In addition, a funnel plot was used to determine the publishing bias. However, due to the limited number of RCTs, interpreting the results was difficult (Figure 8).

## 9. Discussion

Although adherence to a particular treatment plan is essential to getting the best possible outcomes, this fact has, for a long time, been disregarded [3]. Patients who are having this treatment not only need to comply with the treatment regimen's standards but also need to make adjustments to their lives, improve the quality of their meals, and so on. Because of this, the significance of dialysis therapy should be stressed. As a consequence of this, the aid of a nurse, which is normally not difficult to get and is quite affordable, is essential for increasing conformity. According to the findings of this meta-analysis, nursing intervention improved patients' conformity with their dialysis treatments by 15% overall. This finding suggests that nursing intervention enhanced patients' conformity by 15% compared to standard therapy. As a consequence of this, a more extensive dissemination of such an intervention and more serious implementation of it may assist ESRD patients live longer. It has been shown that nursing intervention, which encompasses educational, cognitive, behavioral, and nutritional strategies, may enhance the physical and mental health of patients with ESRD [10, 12–14]. Despite this, the conclusions that may be found in the body of research are contradictory; the impact measurements are unique and cannot be compared. For example, weight and IDWG were utilized as significant outcomes in a number of investigations [13], whilst biomarkers such as phosphorus, Kt/V, or albumin were used in a number of other research studies. In this particular research, we combined a number of different indicators into a single, more comprehensive, clinically relevant, and comparable measurement, which we called dialysis conformity. Furthermore, we discovered through our meta-analysis that preliminary investigation of the effect of various intervention methods revealed no significant differences; however, the ability to draw a conclusion was hindered due to potential bias resulting from cultural and ethical differences, as well as subtle differences in the same category of intervention from different studies. The country disparity was larger, and the intervention's impact was less substantial in China than it was in Europe and the United States (12 vs. 19%). Patients in China may be reluctant to follow treatment plan and lack essential health awareness, and nurses and catechists in China may lack necessary health consciousness, based on the results of this study, in which the western world had a higher than average effect (19 vs. 15%), while China had the opposite (12 vs. 15%). Patients living in countries with a higher standard of living have clearly greater access to a larger variety of medical services and benefits. Additionally, we may see that medical personnel have comprehension and professional abilities, in addition to acceptance and support for the introduction of medical innovations. It may be very challenging to increase people's awareness and desire to participate. However, the Chinese government and the healthcare sectors need to devote more effort to strengthening the educational facilities in order to remove preconceptions against the treatment provided by medical professionals and behaviours toward medical care in general. This can only be accomplished by educating the public about the benefits of receiving treatment from medical professionals.

This meta-analysis does not come free of a number of restrictions (Figure 9). These studies may suffer from communication bias and lack of blinding due to the mathematical translation of symptoms into conformity. This is due to the fact that the nature of the therapies themselves may have the potential to contribute to bias. Second, determining the impact was challenging since various studies used varied numbers of treatments (single, double, or triple), and geographical and climatic conditions made comparisons difficult. Third, the quantity and quality of related studies were restricted, and only a handful could be included. Even if the researcher utilized randomization, one of the nine studies examined found to have a low-balanced baseline.

The most significant advantage of this meta-analysis is that it evaluated the impact of nursing intervention by using a singular outcome, namely, dialysis conformity, which was a very significant clinical signal. Furthermore, a statistically significant summed RD of 15% was discovered. As a result, this meta-analysis provides data and a foundation for improving nursing care for ESRD patients receiving dialysis in everyday clinical practice. Finally, the findings imply that raising people's health awareness and reducing medical personnel deaths is crucial in developing nations like China, which is given as an example here. Given China's large population, this has the potential to be extremely important for global humanity's well-being. A forest plot showing the supplementary RCT analyses of control conformity is shown in Figure 10.

## 10. Patients' Self-Ratings on the Anxiety Scale before and after Nursing Intervention in the Two Groups

Prior to the nursing diagnosis, when the SAS ratings of the participants in two distinct groups were compared to one another, there was no discernible substantial distinction. After an amount of time equal to five months, the patients who took part in the research saw a noticeable decline in their SAS scores, and the differences between the two groups were significant statistically (*p* 0.01). On the other hand, the SAS scores of the patients who served as controls had not changed (*p* > 0.05). The research group's scores were clearly lower than the control group's five months following the nursing intervention, and the differences were statistically significant (see Table 3).

## 11. Patients' Self-Rating Depression Scale Scores before and after Nursing Intervention in Two Groups

When the SAS ratings of the individuals in the 2 categories were compared following the nursing intervention, there was no apparent difference between the groups. After being a part of the research group for a period of four weeks, there was a visible decline in the SDS ratings of the patients, and the variations were statically important (*p* 0.01). On the other hand, the patients who were a part of the management group did not see a statistically significant change in their SDS score (*p* > 0.05). The ratings of the research team were significantly lower than the ratings of the control group five months following the nursing intervention; the group differences were statically important. The research group had received the nursing intervention (see Table 4).

## 12. Baby Results

Skin rashes, concerns about privacy, and illness caused three of the 96 persons who initially volunteered for the study to later withdraw from participation. As a direct and immediate result of this, there were just 93 participants who were successful in completing the entire research project (30 in experimental group 1, 31 in experimental group 2, and 32 in the control group). A three-percent drop in membership was seen throughout the course of the year. According to research using descriptive statistics that was based on the demographic and clinical data of 93 people at the beginning of the study, the following was found to be accurate: 53 (5699%) had an elementary school education or higher; the average age was 6188 (SD 127) years; 69 (7419%) were economically inactive; 70 (7527%) were religious; 69 (7419%) were married; 74 (7957%) had high blood pressure; 40 (4301%) were diabetic; and 53 (5699%) had an elementary school education or higher. 27 of them, which is 2903.3%, suffered from heart disease, and 44 of them, which is 4731.3%, were on hemodialysis for one to 3 years (on average, one to three years). Diabetes was the primary renal ailment in 34 of the people, which is 3.56% of the total. In all, 78 (or 83.87%) of the participants had a dialysis treatment that lasted for four hours or more. The most typical F10-HPS and B1–16 dialyser models were used. The kind of the dialyser used was usually determined by the body weight of the patient. The contributor patients who were underweight usually utilized low-flux (specified as a coefficient of ultrafiltration of less than 30 cc/h. Dialyzer (mmHg), such as B1-16, those with large subjects, and typically, high-throughput (also known as ultrafiltration) systems are used. In dialyser (coefficient > 30 cc/h/mmHg), such as the F10-HPS, 265 (SD 388) cc/min was the average blood flow rate; 53 polysulfone dialysis membrane was utilized by 5761%; 60 (6452%) reported dry skin issues; 18 (or 19%) were presently taking pruritus medication; average duration of pruritus was 4058 months (SD 378). The statistical data for each category are summarized in Tables 5 and 6. The findings revealed that the three groups shared several demographic and dialysis data similarities. On the other hand, in comparison with the other groups, the control group had a much smaller number of persons who were married, and the experimental group 2 had a significantly larger number of participants whose skin was dry (*p* 005). According to the results of multiple regression analysis, there was no significant correlation between pruritus and either married status or dry skin (*p* = 093 and 073, respectively). Therefore, the three groups were assumedly homogenous.

The average total ISS scores for the 93 subjects in terms of current pruritus state were 664 (SD 31) with a range of 135–1483. Pruritus was experienced by 74 (7957%) of the participants in the morning, 74 (7957%) in the afternoon, 80 (8602%) in the evening, and 88 (9462%) in the late evening. A twinge was experienced by 24 (2581%) people, tingling by 23 (2473%) people, and burning by 21 (2258%) people who had pruritus. 35 (3763%) said their pruritus was unpleasant, 21 (2258%) said it was extremely bothersome, and 35 (3763%) said it was terrible.  Table 7 presents the baseline ISS scores for the three groups. Before the baby oil intervention, analysis of variance was done to assess group homogeneity. The ANOVA findings indicated that the three groups had substantially different baseline values for pruritus severity (df = 2, *F* = 1311, *p* 00001). The severity of pruritus in experimental group 1 was substantially greater than in the control group. To compare scores before and after intervention, a paired *t*-test was performed. Significant improvements in pruritus ratings in all three groups (experimental group 1 (*t* = 656, *p* 00001), experimental group 2 (*t* = 1187, *p* 00001), and control group (*t* = 861, *p* 00001) revealed that each group's itching had significantly improved (Table 8). Significant differences in pruritus ratings were found using analysis of variance (df = 2, *F* = 883, *p* = 00003) (Table 9).

## 13. Conclusion

Based on these findings, it is clear that the standard of treatment for end-stage renal disease (ESRD) patients who are on dialysis has to be bolstered. An essential goal of this study was to provide the groundwork for future research on the issue. Traditional nursing care combined with psychological nursing intervention can significantly enhance the psychological states of hemodialysis patients with uremia, lowering anxiety, and sadness levels. Nurses and other health professionals recognize the need to demonstrate that their care is high quality, effective, and also cost-effective. Evaluating nursing interventions helps them evaluate their programs to meet this need.

## Figures and Tables

**Figure 1:** ESDR related factor.

**Figure 2:** The function *f*attains the slope of the secant between *a* and *b* as the derivative at the point *ξ* ∈ (*a*, *b*).

**Figure 3:** Standard deviation concept.

**Figure 4:** An example with the same mean but different standard deviations is provided. The red and blue populations' averages and standard deviations are 100 and 50, respectively.

**Figure 5:** The process flow of the meta-analysis search approach.

**Figure 6:** A plot depicting meta-analyses of randomized controlled trials comparing dialysis adherence in the nursing intervention. Each unit contains a study, and its size is equal to the average treatment effect accuracy of the research. The horizontal line reflects the 95% confidence interval for the outcome measures in each study. The diamond's center reflects the average treatment effect across trials, while the breadth represents the diamond's 95% confidence interval.

**Figure 7:** A forest plot depicting meta-analyses of RCTs comparing dialysis obedience in the control groups.

**Figure 8:** Conformity in a funnel plot (RD).

**Figure 9:** A forest plot showing the supplementary RCT analyses of experimental.

**Figure 10:** A forest plot showing the supplementary RCT analyses of control conformity.

**Table 1:** Intervention protocol.

Stages	Steps
Preparation	(1) Give the patient a hospital gown and a blanket (2) Examine the afflicted region with a medical exam examination light (3) Thoroughly wash your hands (4) Use a thermometer to ensure that the oboe's oil is between 10 and 15 degree Celsius

Execution	(1) Use cooled or unchilled tub oil to relieve itching caused by acute cystitis. (2) Apply either cooled or unchilled baby oil to the affected region if you are experiencing pruritus or excessive dryness. Each application of cold baby oil should only last for fifteen minutes at the most so as to prevent any pain. (3) When one is suffering from roaring itching as a result of pruritus or excessive dryness, the suggested amount of time between applications of cooled baby oil is thirty to sixty minutes.

Conclusion	(1) Participants are free to get dressed and relax for the remainder of the session after using either chilled or unchilled OOb)'oil. (2) It is important to keep track of any changes in the skin or the body (Chen 2006, Chiu & Hsieh 200.S). (3) Once the temperature within the refrigerator has been verified, the baby oil that has been cooled should be placed inside the refrigerator. Baby oil that has not been refrigerated should be kept at room temperature.

Emergency administration for the use of cooled obe'oil	(1) If the patient is experiencing shaking, numbness, or discomfort, you must immediately stop the treatment procedure (2) Check to see if the patient's vital signs are steady and that they are maintained (3) If the patient is complaining of pain, it is imperative that you seek medical attention

**Table 2:** The primary distinguishing features of the nine studies that were published between 2003 and 2016.

Study number	Average of age, years (I/C)	Male/female	Sample size (I/C)	Withdrawal number (I/C)	Intervention (experimental group)	Measurements of outcome	Study design/Jadad score
1	45.6/45.3	56/44	50/50	NA	Educational, psychological, dietary intervention	Conformity	RCT, open (O)/3

2	65.2/63.6	107/113	110/110	12/7	Cognitive, emotional, intervention, behavioral	Conformity weight Conformity IWDG	RCT, O/4 RCT, O/3 RCT, O/3 RCT, O/3 RCT, O/3 RCT, O/3 RCT, O/4

3	61.1/61.2	38/32	35/35	NA NA NA	Educational intervention cognitive, behavioral intervention cognitive, behavioral intervention behavioral intervention educational training	Phosphorus IWDG	RCT, O/3 RCT, O/3

4	49.5/50.01	14/1	8/7	1/1	Diet education	Conformity conformity	RCT, O/4 RCT, O/3 RCT, O/3 RCT, O/3 RCT, O/3 RCT, O/3 RCT, O/4

5	55.9/58.2	46/33	39/40	4/3	Cognitive behavior therapy	Conformity weight conformity IWDG IWDG	RCT, O/3 RCT, O/3

6	56.9/58.1	78/41	61/58	NA	Educational, psychological, dietary intervention	Phosphorus IWDG	RCT, O/4 RCT, O/3 RCT, O/3 RCT, O/3 RCT, O/3 RCT, O/3 RCT, O/4

7	NA 56.1/52.5	28/36	32/32	NA	Cognitive, emotional, behavioral intervention	Conformity conformity	RCT, O/3 RCT, O/3

8	46.6/46.9	24/39	35/35	12/7	Educational intervention cognitive, behavioral intervention cognitive, behavioral intervention behavioral intervention educational training	Conformity weight conformity IWDG IWDG	RCT, O/4 RCT, O/3 RCT, O/3 RCT, O/3 RCT, O/3 RCT, O/3 RCT, O/4

9	65.2/63.6	38/18	29/27	NA	Diet education	Phosphorus IWDG	RCT, O/3 RCT, O/3

**Table 3:** The SAS scores of uremia patients on hemodialysis in two groups.

Group	Cases		SAS
Control group	33	Before treatment After treatment	57.0 ± 4.1 56.5 ± 3.8
Research group	27	Before treatment After treatment	56.8 ± 5.0 47.6 ± 4.8

**Table 4:** The SDS scores of uremia patients on hemodialysis in two groups.

Group	Cases		SDS
Control group	33	Before treatment After treatment	49.9 ± 1.7 51.5 ± 2.0
Research group	27	Before treatment After treatment	54.2 ± 1.9 46.8 ± 2.1′

**Table 5:** Analyses of the demographic and medical baseline data for the experimental groups 1 and 2 as well as the control group were performed.

Items	Experimental group 1 (*n* = 30)	Experimental group 1 (*n* = 31)	Experimental group 1 (*n* = 32)	*p*
Male	18 (56.67)	17 (52.62)	22 (69.75)	0.25

Female	14 (43.33)	16 (49.38)	10 (31.35)

Age (years)				
17–63	17 (54.31)	13 (39.71)	18 (56.20)	0.19
64–75	9 (27.71)	17 (52.61)	8 (26.10)	
Above 75	7 (21.01)	4 (9.71)	6 (19.80)	

Degree of education				
Basic	18 (64.34)	22 (68.75)	13 (41.73)	0.07
Junior	5 (14.34)	5 (13.91)	6 (19.65)	
Secondary school	6 (24.34)	7 (18.34)	13 (41.73)	

Occupation				
Working	8 (24.34)	10 (28.02)	8 (26.10)	0.88
Not working	24 (86.68)	23 (71.98)	24 (76.10)	

Relationship status				
Married	28 (97.68)	29 (91.31)	24 (76.10)	0.04^*∗*^
Single	2 (34.34)	4 (10.65)	8 (26.10)	

Religion				
Yes	23 (74.34)	24 (75.16)	25 (79.23)	0.88
No	9 (27.68)	9 (26.82)	7 (22.98)	

**Table 6:** Experimental group 1, experimental group 2, and control group (*n* = 93) hemodialysis data.

Items	*n* (%)	Average (SD)	*n* (%)	Average (SD)	*n* (%)	Average (SD)	*p*
Total time spent on hemodialysis (months)		74.03 (52.96)		61.04 (42.15)		76.51 (57.83)	0.87

Dialysis-related kidney disease in its most basic form							
HTN	4 (14.34)		3 (9.69)		4 (14.52)		0.26
DM	15 (45.65)		8 (28.04)		11 (34.38)		
CGN	6 (21.01)		7 (25.82)		8 (25.00)		
SLE	4 (14.34)		5 (17.03)		2 (6.25)		
Others	3 (7.77)		7 (18.45)		7 (21.88)		

Duration of dialysis (hours)							
3.0	0 (0.01)		3 (7.43)		0 (0.01)		0.06
3.5	0 (0.01)		3 (9.68)		1 (7.26)		
4.0	28 (91.0)		24 (81.64)		27 (82.26)		
4.5	4 (10.01)		2 (4.24)		5 (13.51)		

Dialysis flow rate (cc/min)		270.00 (31.06)		261.29 (41.61)		272.45 (42.41)	0.32

Dialysis membrane							
PMMA	5 (14.34)		6 (21.59)		3 (6.44)		0.06
Polysulf	14 (47.68)		18 (62.28)		21 (65.53)		
Others	13 (41.01)		4 (15.12)		8 (29.01)		

Dry skin							
Yes	17 (54.34)		27 (87.10)		18 (54.12)		0.01^*∗*^
No	15 (56.77)		4 (12.90)		16 (47.87)		

Antihistamine							
Yes	5 (21.01)		4 (12.90)		9 (25.01)		0.48
No	25 (81.00)		27 (87.10)		25 (75.01)		

The total time spent itching (months)		53.83 (49.01)		31.19 (27.24)		36.26 (31.61)	0.05

^*∗*^ *p* < 0.05.

**Table 7:** Experimental group 1, experimental group 2, and control group (*n* = 93) baseline itch severity scale.

Items	STD group experiment 1	STD group experiment 2	STD control group
Total	7.76 (3.19)	7.65 (2.66)	4.65 (2.33)
Frequency	0.48 (0.23)	0.55 (0.25)	0.35 (0.15)
Itch definition	0.35 (0.26)	0.24 (0.25)	0.09 (0.15) affected body surface area
The influence on sexual attraction 0.10 (0.31)	0.07 (0.26)	0.04 (0.19) effect on sleep	0.42 (0.32)
Total	7.76 (3.19)	7.65 (2.66)	4.65 (2.35)
Frequency	0.48 (0.23)	0.55 (0.25)	0.37 (0.17)
Itch definition	0.35 (0.26)	0.24 (0.25)	0.09 (0.15) affected body surface area
The influence on sexual attraction 0.10 (0.31)	0.07 (0.26)	0.04 (0.19) effect on sleep	0.42 (0.32)

**Table 8:** Pretest and posttest itch severity scale ratings for each group (*n* = 93).

Entry	Group experiment 1			Group experiment 2			Control group		
	(Std)	*t*	*p*	(Std)	*t*	*p*	(Std)	*t*	*p*
Difference frequency	3.82 (3.18)	6.5	<0.01^*∗*^	3.12 (2.43)	—12.77	<0.01^*∗*^	1.05 (2.48)	8.40	<0.01^*∗*^
Pre	0.39 (0.21)	5.29	<0.01^*∗*^	0.55 (0.25)	6.88	<0.01^*∗*^	0.34 (0.17)	3.41	<0.01^*∗*^
Post	0.29 (0.18)			0.34 (0.21)			0.25 (0.17)		

Sensibility									
Pre	0.35 (0.24)	6.11	<0.01^*∗*^	0.24 (0.25)	3.71	<0.01^*∗*^	0.09 (0.15)	0.27	0.88
Post	0.08 (0.11)			0.12 (0.19)			0.09 (0.14)		

Area									
Pre	0.53 (0.24)	3.32	<0.01^*∗*^	0.63 (0.28)	3.24	<0.01^*∗*^	0.42 (0.28)	0.69	0.42
Post	0.33 (0.29)	2		0.41 (0.31)			0.37 (0.31)		

Level									
Pre	0.54 (0.1)	5.22	<0.01^*∗*^	0.52 (0.18)	6.78	<0.01^*∗*^	0.39 (0.18)	1.41	0.13
Post	0.34 (0.18)			0.33 (0.16)			0.32 (0.19)		

Emotion									
Pre	0.19 (0.16)	4.36	<0.01^*∗*^	0.15 (0.17)	1.08	0.29	0.08 (0.22)	1.23	0.23
Post	0.08 (0.12)			0.11 (0.15)			0.04 (0.13)		

Sex									
Pre	0.11 (0.32)	1.90	0.08	0.07 (0.26)	1.42	0.16	0.02 (0.19)	—	—
Post	0.01 (0.01)			0.01 (0.01)			0.02 (0.19)		

Sleep									
Pre	0.42 (0.32)	3.81	<0.01^*∗*^	0.45 (0.25)	5.96	<0.01^*∗*^	0.21 (0.22)	2.13	0.06
Post	0.24 (0.27)			0.24 (0.28)			0.11 (0.19)		

^*∗*^ *p* < 0.05.

**Table 9:** A comparison of the changes in itching severity scale scores that occurred before and after the test for each of the three groups (*n* = 93).

Group (n)	(Std)	*P* from ANOVA	Orders
Experiment 1 (30)	3.51	0.0005^*∗*^	Experiment 1
Experiment 2 (31)	3.11 (2.44)		Experiment 2
Control (32)	1.04 (2.47)		

## Data Availability

No data were used to support this study.
